RETRACTED

# Influences of Antithrombotic Elastic Socks Combined with Air Pressure in Reducing Lower Extremity Deep Venous Thrombosis for Patients Undergoing Cardiothoracic Surgery

**DOI:** 10.1155/2022/1338214

**Published:** 2022-09-05

**Authors:** Weihong Fu, Qun Zhang, Xuemei Sun, Yan Gu

**Affiliations:** ^1^Department of Thoracic Surgery, Affiliated Hospital of Nantong University, Nantong, 226001 Jiangsu, China; ^2^Department of Cardiovascular Surgery, Affiliated Hospital of Nantong University, Nantong, 226001 Jiangsu, China; ^3^Department of Surgery, Affiliated Hospital of Nantong University, Nantong, 226001 Jiangsu, China

## Abstract

This study was designed to investigate the application and therapeutic effect of antithrombotic elastic socks combined with air pressure in the prevention of lower extremity deep venous thrombosis in patients undergoing cardiothoracic surgery. Sixty patients in cardiothoracic surgery of our hospital from January 2019 to December 2020 were randomly divided into a study group and control group. The control group was treated with routine treatment intervention. Based on routine treatment intervention, the study group was treated with antithrombotic elastic socks combined with pneumatic treatment intervention. The activated partial thromboplastin time (APTT), thrombin time (TT), femoral venous blood flow velocity of both lower limbs, and the incidence of lower extremity deep venous thrombosis (LEDVT), postoperative lower extremity swelling, inflammatory factors, and satisfaction were measured. After intervention, APTT (31.74 ± 1.15 s) and TT (14.58 ± 0.24 s) in the study group were higher than those in the control group APTT (25.13 ± 1.14 s) and TT (12.14 ± 0.23 s) (*P* < 0.05). The left lower limb femoral vein blood flow velocity and the right lower limb femoral vein blood flow velocity in the study group were better than those in the control group (*P* < 0.05). The incidence of postoperative lower limb swelling and deep vein in the study group was lower than that in the control group (*P* < 0.05). Serum tumor necrosis factor alpha and interleukin-6 concentrations in the study group were lower than those in the control group (*P* < 0.05). The satisfaction rate of patients in the study group (93.33%) was significantly higher than that in the control group (70.00%) (*P* < 0.05). In conclusion, after cardiothoracic surgery, antithrombotic elastic socks combined with air pressure can significantly reduce the incidence of LEDVT by improving patients' coagulation function, reducing inflammatory reaction. It is worthy of popularization and application in relevant surgery.

## 1. Introduction

Venous thrombosis is often caused by trauma and surgery, and abnormally coagulated blood can lead to partial or even complete obstruction of vascular lumen. Lower extremity deep venous thrombosis (LEDVT) is one of the most common surgical complications in clinic [1]. Surgical treatment is one of the main treatment methods for lesions in the esophagus, lungs, mediastinum, and other parts [2]. Cardiothoracic surgery is a clinical department mainly for major surgical treatment, mostly for elderly patients, and the surgical site involves important organs of the human body. The operation is complicated and traumatic, and the postoperative recovery is slow, which requires long-term bed rest and more complications. Cardiothoracic surgery, the patient needs to stay in bed for a long time after operation, resulting in slow and blocked blood reflux, which is very easy to be complicated with deep venous thrombosis of lower limbs [3]. LEDVT can lead to lower limb swelling, pain and other symptoms, and even fatal pulmonary embolism, threatening the life and health of patients. At present, the methods to prevent deep venous thrombosis mostly take drugs or physical methods to reduce the viscosity of blood and promote the blood circulation of lower limbs. However, it is difficult to control the dosage of drug prevention, which is easy to cause postoperative bleeding [4, 5]. Various physical prevention methods, including postoperative massage and electrical stimulation of calf muscles, are sometimes difficult to achieve the expected effect due to difficult control and large individual differences. Similarly, muscle electrical stimulation is difficult for most patients to accept because it increases the discomfort of postoperative patients.

RETRACTED

The antithrombotic elastic socks are designed according to the characteristics of human physiological function, and the pressure decreases gradually from the distal ankle to the proximal end. The venous blood of the distal leg can be pumped back to the heart to improve the blood circulation of both lower limbs. The antithrombotic elastic socks cover the foot to the knee, and the feet expose the toes, which is the intervention to shrink calf muscles and prevent venous filling. Meanwhile, the antithrombotic elastic socks are convenient to observe the blood circulation and allow blood to flow back to the heart through progressive pressure [6, 7]. Pneumatic therapy is a kind of “physiological pump” simulating artificial massage, which compresses the muscles of both lower limbs by rapidly inflating and deflating the air bag in a short time, so as to accelerate the blood reflux in the venous cavity, accelerate the venous blood circulation, and rapidly increase the blood perfusion and oxygenation speed [8, 9]. Pneumatic therapy can increase the rate of venous return to enhance the blood circulation of the lower limbs and reduce the incidence of LEDVT [10].

RETRACTED

The purpose of this study was to explore the application and therapeutic effect of antithrombotic elastic socks combined with pneumatic therapy in the prevention of lower extremity deep venous thrombosis in patients undergoing cardiothoracic surgery.

## 2. Data and Methods

### 2.1. General Information

A total of 60 patients admitted to cardiothoracic surgery from January 2019 to December 2020 were randomly divided into a study group (*n* = 30) and control group (*n* = 30). This study was approved by the medical ethics committee of the hospital and obtained the consent of the selected patients and their families, and all patients signed the informed consent form. Inclusion criteria were as follows: all patients need thoracic surgery, no surgical contraindications, and good compliance. Exclusion criteria were as follows: patients with coagulation dysfunction, heart and liver dysfunction, or cognitive impairment.

There was no significant difference in gender, age, height, weight, operation time, and other general data between the two groups (*P* > 0.05), as shown in Table 1.

### 2.2. Intervention Methods

*Control group*: routine nursing prevention was adopted. Before operation, nurses explained the principle and risk of lower extremity deep venous thrombosis to patients and their families and made a comprehensive evaluation, explain the methods and significance of prevention of postoperative deep venous thrombosis of lower limbs, and inform the patients of perioperative diet precautions and the significance of getting out of bed as soon as possible after operation. After operation, patients are encouraged to get out of bed early and step by step. The whole process must be completed under the supervision and guidance of nurses or accompanied by family members. If the patient is not fit to get out of bed, the nurse shall assist the patient in passive exercise after the condition is stable. Specific methods are as follows: start from the distal small joints of both lower limbs; perform flexion, extension, and lifting in the order from toe to hip joint, three times a day, 20 minutes each time; and teach the family members.

*Study group*: on the basis of the control group, medical elastic socks and pneumatic therapeutic instrument were used for prevention. (1) Before operation, measure the thinnest and coarsest circumference of the patient's lower leg, and select medical elastic socks of appropriate specification and length. The nurse shall help to wear medical elastic socks to ensure that the toes are exposed. Pay close attention to the tightness of medical elastic socks, the skin temperature on the back of the foot, and the pulsation of the artery on the back of the foot. During the period, pay attention to personal hygiene and replace and clean them frequently. (2) Use of pneumatic therapeutic instrument: the patient takes a flat lying position, puts his lower limbs into the sleeve of pneumatic therapeutic instrument, and the sole of the foot reaches the bottom of the sleeve with appropriate tightness. The pressure is set to 25-180 mmHg (1 mmHg = 0.133 kPa). According to the manufacturer's instructions, set the ankle 45 mmHg, lower leg 40 mmHg, and thigh 30 mmHg to ensure the blood flow to the proximal heart. When inflating, start from the air bag at the distal end of the lower limb and gradually inflate to the proximal end until the air bag at the root of the thigh is inflated and all the air bags in the sleeve are automatically and slowly vented [11]. The above methods were performed twice a day for 30 minutes each time until the fifth day after operation. In addition to bathing or taking off and replacing in time in case of pollution, it is necessary to keep wearing medical elastic socks until the fifth day after operation, including functional exercise in bed and out of bed activities. In the course of treatment, closely observe the patient's reaction, and stop treatment immediately in case of complexion change, chest tightness, palpitation, etc.

RETRACTED

### 2.3. Observation Indicators

1. Coagulation function index: 3 mL of peripheral venous blood sample was collected from each patient before and after intervention. QLabs Electrometer (Micropoint Biotechnologies, Guangdong, China) was used to test the samples for activated partial thromboplastin time (APTT) and thrombin time (TT)
2. Femoral vein blood flow velocity of both lower limbs: the femoral vein blood flow velocity of both lower limbs of the two groups was measured before and after the intervention
3. The incidence of LEDVT in the two groups was recorded
4. Lower extremity deep venous thrombosis: the peripheral diameters of lower leg and thigh were measured 1 day before operation and 1-3 days after operation, and the postoperative lower limb swelling of the two groups was comprehensively evaluated. Deep veins of lower limbs: the same doctor with ultrasonic diagnosis qualification shall detect the deep veins of both lower limbs of the two groups by ultrasonic detection on the first day before operation and the first to third days after operation, so as to determine whether there is lower limb venous thrombosis
5. Tumor necrosis factor-*α* (TNF-*α*) and interleukin-6 (IL-6) were detected by ELISA as previously reported [12]. The kit was produced by Shanghai Kanglang Biotechnology Co., Ltd.
6. Patients' satisfaction was evaluated by self-made questionnaire at discharge, including nursing staff's professional level, comfort, and working attitude. The full score is 100 points. A score of 90-99, 75-89, and less than 75 points meant that the patients are very satisfied, satisfied, and dissatisfied, respectively.

RETRACTED

### 2.4. Statistical Analysis

The SPSS v20.0 software (IBM, USA) was used for data analysis. The comparison between the two groups of data adopts *t*-test, and all measurement data are expressed by mean ± standard deviation (mean ± SD). *P* < 0.05 is considered as the difference which is statistically significant.

## 3. Results

### 3.1. Comparison of Coagulation Function Indexes between the Two Groups before and after Intervention

Before the intervention, there was no significant difference between APTT and TT in the two groups (*P* > 0.05). After the intervention of different modes, APTT and TT in the study group were significantly better than those in the control group (*P* < 0.05), as shown in Table 2.

### 3.2. Comparison of Blood Flow Velocity of the Femoral Vein of Both Lower Limbs between the Two Groups before and after Intervention

Before the intervention, there was no significant difference in the blood flow velocity of the lower limb femoral vein between the two groups (*P* > 0.05). After the intervention of different modes, the blood flow velocity of the lower limb femoral vein in the study group was significantly higher than that in the control group (*P* < 0.05), as shown in Table 3.

### 3.3. Comparison of Postoperative LEDVT Incidence between the Two Groups

There were 8 cases of postoperative lower limb swelling and 6 cases of deep venous thrombosis in the control group, with the incidence of about 26.67% and 20%. There was 1 case of postoperative lower limb swelling and 0 case of deep venous thrombosis in the study group, with the incidence of about 3.33% and 0.00%, which was significantly lower than that in the control group (*P* < 0.05), as revealed in Table 4.

### 3.4. Comparison of Serum Inflammatory Factor Expression between the Two Groups

Before the intervention, there was no significant difference between the serum inflammatory factor indexes TNF-*α* and IL-6 in the two groups (*P* > 0.05). After the intervention of different modes, the TNF-*α* and IL-6 in the study group were significantly lower than those in the control group (*P* < 0.05), as shown in Table 5.

### 3.5. Comparison of Patients' Satisfaction with Treatment between the Two Groups

The overall satisfaction rate of the study group was 93.33%, significantly higher than 70.00% of the control group (*P* < 0.05), as shown in Table 6.

RETRACTED

## 4. Discussion

Deep venous thrombosis (DVT) is one of the most common perioperative complications, which can lead to pulmonary embolism and can even be life-threatening. In patients with pulmonary embolism, 90% of the thrombus is caused by the falling off of the deep venous thrombosis of the lower limbs and entering the pulmonary artery through the blood circulation [13]. With the continuous improvement of diagnostic technology, the incidence of the disease shows an increasing trend, however. The occult onset and delayed diagnosis of deep venous thrombosis may delay the best time of treatment. Therefore, it is of great significance to take active measures to prevent deep venous thrombosis [14].

The surgical trauma of cardiothoracic surgery is generally large and the postoperative stay in bed is long, suggesting that the prevention of postoperative deep venous thrombosis is particularly important. In this study, the average ages of the two groups were 64.63 ± 5.44 years and 64.93 ± 5.68 years. Most of the patients are elderly patients, with decreased cardiac output, slow blood flow, and even stasis. In addition, the patient fasted for a long time before operation, the body volume was relatively insufficient, and the blood viscosity increased, which increased the risk of postoperative deep venous thrombosis. Meanwhile, elderly patients with reduced postoperative activity and long resting time can cause slow blood flow; intraoperative operation and deep vein catheterization can cause vascular injury.

The principle of antithrombotic elastic socks is to accelerate the speed of venous blood circulation, reduce venous blood stasis, and then promote the blood circulation of the lower limb veins, which can continuously and effectively prevent lower limb deep venous thrombosis in patients undergoing cardiothoracic surgery. Barotherapeutic instrument, as a noninterventional therapeutic instrument, has the same principle of action as manual massage. The mechanical pump is used to quickly inflate and exhaust the air bag on the sleeve in a very short time to squeeze the limbs, which can accelerate the blood circulation in the veins of the limbs and improve the blood perfusion and oxygenation of the limbs [15, 16]. Compared with manual massage, pneumatic therapeutic instrument has the advantages of simple operation, small individual difference, and no influence of body position. The research shows that the design of different pressure gradient can increase the blood flow rate and shorten the recovery time of skin temperature, which is of positive significance to prevent the occurrence of deep venous thrombosis after shell surgery. In addition, this operation can also reduce the workload of its nurses, so as to devote more energy to observing the changes of the disease and perioperative nursing, and significantly improve the satisfaction of patients with nursing work. By comparing the postoperative lower limb swelling, the incidence of postoperative deep venous thrombosis, hospitalization time, and hospitalization expenses between the two groups, we found that medical elastic socks combined with pneumatic therapeutic instrument can significantly improve the postoperative recovery, shorten the hospitalization time, save medical expenses, and improve the postoperative quality of life.

RETRACTED

The results showed that before the intervention, there was no significant difference between APTT and TT, as well the blood flow velocity of the lower limb femoral vein in the two groups (*P* > 0.05). However, after the intervention of different modes, APTT and TT in the study group were significantly better than those in the control group (*P* < 0.05). Meanwhile, the blood flow velocity of the femoral veins in both lower limbs in the study group was significantly faster than that in the control group (*P* < 0.05). The reasons may be as follows: (1) the gradient pressure effect of antithrombotic elastic socks; (2) the compression frequency and inflation time were adjusted in time, and the air pressure gradually intervened in both lower limbs from the distal end to proximal end, so as to improve the hemodynamic indexes. Studies have shown that barotherapy can improve the biological activity of plasmin, promote fibrinolysis, inhibit the activation of procoagulant substances, and prevent coagulation factors from adhering to the intima of blood vessels. Our study showed that the incidence of postoperative lower limb swelling and deep vein in the study group was lower than that in the control group (*P* < 0.05). IL-6 and TNF-*α* are important inflammatory factors that mediate the process of platelet aggregation [17]. Some scholars believe that inflammatory factors may play key roles in the occurrence and development of LEDVT [18]. Consistently, our study found that before the intervention, there was no significant difference between the serum inflammatory factor indexes TNF-*α* and IL-6 in the two groups (*P* > 0.05). After the intervention of different modes, the TNF-*α* and IL-6 in the study group were significantly lower than those in the control group (*P* < 0.05). The decrease of the IL-6 and TNF-*α* expression indirectly suggested that the risk of LEDVT also decreases. In addition, our research demonstrated that the overall satisfaction rate of the study group was 93.33%, significantly higher than 70.00% of the control group (*P* < 0.05). All the above findings indicated that the use of antithrombotic elastic socks combined with pneumatic treatment may play a good effect in the prevention of LEDVT after cardiothoracic surgery.

RETRACTED

## 5. Conclusion

The application of antithrombotic elastic socks combined with pneumatic therapy in perioperative patients of cardiothoracic surgery can effectively reduce the incidence of lower extremity deep venous thrombosis, improve patients' coagulation function, and improve satisfaction, which is worthy of clinical application.

## Figures and Tables

**Table 1:** Comparison of general data between the two groups.

Groups	*n*	Age (years)	Gender (*n*)		Height (cm)	Body weight (kg)	Operation time (min)
			Male	Female			
Control group	30	64.63 ± 5.44	18	12	162.86 ± 7.62	66.77 ± 11.53	194.52 ± 44.63
Study group	30	64.93 ± 5.68	15	15	462.66 ± 9.12	69.63 ± 10.40	176.71 ± 43.52
*P*		>0.05	>0.05		>0.05	>0.05	>0.05

**Table 2:** Comparison of coagulation function indexes between the two groups before and after intervention (s, *x* ± *s*).

Groups	*n*	APTT		TT	
		Before intervention	After intervention	Before intervention	After intervention
Control group	30	20.83 ± 1.44	25.13 ± 1.14	11.08 ± 0.31	12.14 ± 0.23
Study group	30	20.80 ± 1.45	31.74 ± 1.15	11.12 ± 0.27	14.58 ± 0.24
*t*		0.085	20.105	0.441	32.062
*P*		>0.05	<0.05	>0.05	<0.05

**Table 3:** Comparison of blood flow velocity of the femoral vein of both lower limbs between the two groups before and after intervention (cm/s, *x* ± *s*).

Groups	*n*	Left lower limb (cm/s, *x* ± *s*)		Right lower limb (cm/s, *x* ± *s*)	
		Before intervention	After intervention	Before intervention	After intervention
Control group	30	14.08 ± 3.31	16.19 ± 4.02	14.06 ± 3.20	16.13 ± 4.21
Study group	30	14.11 ± 3.21	19.50 ± 5.03	14.01 ± 3.01	19.20 ± 4.18
*t*		0.039	3.402	0.066	2.722
*P*		>0.05	<0.05	>0.05	<0.05

**Table 4:** Comparison of postoperative lower limb swelling and deep venous thrombosis between the two groups (cases (%)).

Groups	*n*	Postoperative lower limb swelling	Deep venous thrombosis
Control group	30	8 (26.67)	6 (20.00)
Study group	30	1 (3.33)	0 (0.00)
*χ* ^2^		6.40	6.67
*P*		<0.05	<0.05

**Table 5:** Comparison of serum inflammatory factors between the two groups (*x* ± *s*).

Groups	TNF-*α* (ng/mL)		IL-6 (pg/mL)	
	Before intervention	After intervention	Before intervention	After intervention
Control group	2.86 ± 0.30	1.59 ± 0.21	24.65 ± 2.13	15.29 ± 0.95
Study group	2.81 ± 0.24	1.04 ± 0.32	26.65 ± 2.21	9.34 ± 0.88
*t*	0.668	5.241	0.012	6.214
*P*	>0.05	<0.05	>0.05	<0.05

**Table 6:** Comparison of patient satisfaction between the two groups (*n* (%)).

Groups	*n*	Very satisfied	Satisfied	Dissatisfied	Satisfaction rate
Control group	30	8 (26.67)	11 (36.67)	11 (36.67)	21 (70.00)
Study group	30	16 (53.33)	12 (40.00)	2 (6.67)	28 (93.33)
*χ* ^2^					5.269
*P*					<0.05

RETRACTED

## Data Availability

Data generated during the study can be obtained from the corresponding author under reasonable request.
